# Exploring the Mechanism of Curcumin on Retinoblastoma Based on Network Pharmacology and Molecular Docking

**DOI:** 10.1155/2022/2407462

**Published:** 2022-07-19

**Authors:** Chengfu Wu, Wenli Zheng, Jifa Zhang, Xingping He

**Affiliations:** ^1^Ophthalmology Department, Affiliated Hospital of Panzhihua University, Panzhihua 617099, Sichuan, China; ^2^Oncology Department, Panzhihua Central Hospital, Panzhihua 617099, Sichuan, China

## Abstract

**Background:**

Curcumin shows great effects of inhibiting tumor cell proliferation, inducing apoptosis, inhibiting tumor metastasis, and inhibiting angiogenesis on a variety of tumors. However, the biological activity and possible mechanisms of curcumin in the treatment of retinoblastoma have not been fully elucidated. This study explored the potential therapeutic targets and pharmacological mechanisms of curcumin against retinoblastoma based on network pharmacology and molecular docking.

**Methods:**

The genes corresponding to curcumin targets were screened from the HERB, PharmMapper, and SwissTargetPrediction databases. Protein-protein interaction (PPI) networks were constructed for the intersecting targets in the STRING database. Cytoscape 3.7.0 was used for network topology analysis and screening of important targets. *R* 4.1.0 software was used for Gene Ontology (GO) function enrichment and Kyoto Encyclopedia of Genes and Genomes (KEGG) enrichment analysis of intersection targets. The molecular structures of curcumin and core target proteins were obtained from PubChem and PDB databases, and the two were preprocessed and molecularly docked using AutoDockTools and PyMOL software.

**Results:**

Through network data mining, we obtained 504 curcumin targets and 966 retinoblastoma disease targets, and 44 potential targets for curcumin treatment of retinoblastoma were obtained by mapping. Three core targets were obtained from network topology analysis. 462 biological processes, 21 cellular compositions, and 34 molecular functions were obtained by GO enrichment analysis. KEGG pathway analysis revealed 94 signaling pathways, mainly involving chemical carcinogenesis-receptor activation, chemical carcinogenesis-reactive oxygen species, viral carcinogenesis, Th17 cell differentiation, etc. The molecular docking results indicated that the binding energy of curcumin to the core targets was less than 0 kJ mol^−1^, among which the binding energy of RB1 and CDKN2A to curcumin was less than −5 kJ mol^−1^ with significant binding activity.

**Conclusion:**

Based on molecular docking technology and network pharmacology, we initially revealed that curcumin exerts its therapeutic effects on retinoblastoma with multitarget, multipathway, and multibiological functions, providing a theoretical basis for subsequent studies.

## 1. Introduction

Retinoblastoma is the most common intraocular malignancy in children, which accounts for 2.5% to 4% of all childhood cancers and has an incidence of 1/18,000 to 1/14,000 [1]. Poor treatment may lead to blindness or death. In order to realize early diagnosis and treatment of retinoblastoma and to reduce the mortality of retinoblastoma, it is particularly important to find the key genes for retinoblastoma. For patients with retinoblastoma, the development of new natural compounds and the search for new therapeutic targets are necessary.

Curcumin is a yellow phenolic pigment with low toxicity, wide medicinal source and low price extracted from the rhizome of Curcuma longa of the ginger family, such as turmeric and tulip, which has a wide application prospect and value in clinical treatment [2, 3]. Curcumin shows great effects of inhibiting tumor cell proliferation, inducing apoptosis, inhibiting tumor metastasis, and inhibiting angiogenesis on a variety of tumors [4–6]. Domestic and foreign scholars have carried out some studies on the effect of curcumin on retinoblastoma [7]. However, traditional Chinese medicine treatment of diseases is based on the mechanism of action of multitarget and multipathway, and there is a relative lack of research in systematically elucidating the action targets and molecular mechanisms of curcumin in the treatment of retinoblastoma, which requires the application of big data to explore the existing target pathways related to curcumin and retinoblastoma.

Network pharmacology is a systems biology approach to study the development of diseases, understand drug-organism interactions, and guide new drug discovery. Therefore, this study aims to investigate the targets and pathways of curcumin and its possible molecular mechanisms of action in the treatment of retinoblastoma by using network pharmacology and molecular docking methods and to provide a reference basis for subsequent studies. The study scheme design is shown in Figure 1.

## 2. Materials and Methods

### 2.1. Screening of Potential Targets of Curcumin for the Treatment of Retinoblastoma

We obtained validated and predicted targets for curcumin via the HERB (http://herb.ac.cn/), PharmMapper (http://www.lilab-ecust.cn/pharmmapper/), and SwissTargetPrediction (http://www. swisstargetprediction.ch/?) databases. Download microarray data GSE24673, GSE97508, and GSE110811 for retinoblastoma from the GEO database (https://www.ncbi.nlm.nih.gov/) and screen for differentially expressed genes using the GEO2R online tool (adj.*P* < 0.05, |logFC|>2) (Table 1). The above retrieved curcumin action targets were mapped to retinoblastoma disease targets to obtain potential targets of curcumin for retinoblastoma treatment.

### 2.2. Protein-Protein Interaction Network Construction, Analysis, and Core Gene Screening

Protein-protein interaction (PPI) networks were constructed using the online database STRING (https://string-db.org/), and TSV format files were saved, which were imported into Cytoscape 3.7.0 software, and the Cyot NCA plug-in was used to further analyze the topology of the regulatory network and screen out the core target genes.

### 2.3. Enrichment Analysis

To explore the core functional and biological pathways associated with curcumin treatment of retinoblastoma, we performed Gene Ontology (GO) function enrichment and Kyoto Encyclopedia of Genes and Genomes (KEGG) pathway analysis using the ClusterProfiler package in *R* 4.1.0 software. The GO functional enrichment analysis and KEGG pathway enrichment analysis screening conditions were set as *P* < 0.05, *q* < 0.05.

### 2.4. Molecular Docking Verification

The core target genes screened by topological analysis were molecularly docked to curcumin. The protein 3D maps of the core target genes were downloaded from the PDB database (https://www.rcsb.org/). Also, download the 3D structure of the curcumin molecule from the PubChem database (https://pubchem.ncbi.nlm.nih.gov/) and convert the format using Open Babel software. With the help of AutoDockTools, the molecular structure of curcumin was optimized, the structure of core gene protein was dehydrated and hydrogenated, and the molecular and protein preservation format was changed to PDBQT format. Molecular docking verification was performed using Auto Dock Vina software, and finally the obtained results were visualized using PyMOL.

## 3. Results

### 3.1. Targets of Curcumin in the Treatment of Retinoblastoma

504 curcumin targets were retrieved from the HERB, PharmMapper, and SwissTargetPrediction databases. The 966 differentially expressed genes of retinoblastoma were screened by GEO2R from three gene chips, GSE24673, GSE97508, and GSE110811. After mapping the curcumin targets to the retinoblastoma targets, 44 intersecting targets were obtained (Figure 2), which were predicted as potential targets for curcumin treatment of retinoblastoma.

### 3.2. GO Functional Enrichment Analysis and KEGG Pathway Enrichment Analysis

The *R* 4.1.0 software was used to analyze the biological processes and molecular functions of the intersecting targets involved in retinoblastoma and to investigate the possible molecular mechanisms of curcumin in the treatment of retinoblastoma. The GO functional enrichment analysis yielded 517 entries, including 462 for Biological Process, 21 for Cellular Component, and 34 for Molecular function. The results were ranked in order of significance, and the top 10 entries for each type of analysis were selected for visualization in *R* software (Figure 3). The biological process mainly involved the regulation of DNA-binding transcription factor activity, peptidyl-tyrosine phosphorylation, peptidyl-tyrosine modification, histone phosphorylation, etc. Cellular Component mainly involved RNA polymerase II transcription regulator complex, chromosome, centromeric region, microtubule-associated complex, spindle microtubule, etc. Molecular function mainly involved protein serine/threonine kinase activity, RNA polymerase II-specific DNA-binding transcription factor binding, DNA-binding transcription factor binding, etc. KEGG pathway enrichment analysis screened 94 signaling pathways (*P* < 0.05) and visualized the top 30 pathways (Figure 4). The main pathways involved were chemical carcinogenesis-receptor activation, chemical carcinogenesis-reactive oxygen species, viral carcinogenesis, Th17 cell differentiation, etc.

### 3.3. PPI Network Construction, Analysis, and Core Gene Screening

The intersection targets were imported into the STRING database to obtain a total of 44 protein nodes for the PPI network, save the PPI network map (Figure 5) with TSV format files, and import the files into Cytoscape 3.7.0 software. Cytoscape 3.7.0 software plug-in CytoNCA calculated the Betweenness Centrality (BC), Closeness Centrality (CC), Degree Centrality (DC), and Eigenvector Centrality (EC) of 44 intersecting target proteins. The calculated median values of BC, CC, DC, and EC were 16.59, 0.46, 7, and 0.15, respectively. A total of 9 target proteins with parameters greater than the median value were filtered to create a sub-network (Figure 6). The second time, BC, CC, DC, and EC of 9 target proteins in the sub-network were calculated. The median values of BC, CC, DC, and EC were 15.7, 0.73, 5, and 0.34, respectively. A total of 3 target proteins with parameters greater than the median value were obtained and the network was created (Figure 6). The three target proteins were the key target proteins of curcumin for the treatment of retinoblastoma.

### 3.4. Docking Results Analysis

We selected the core targets, including RB1, STAT3, and CDKN2A, for molecular docking with curcumin. The results showed that curcumin has a good affinity with RB1, STAT3, and CDKN2A, and the docking results were visualized by PyMOL software (Figure 7 and Table 2).

## 4. Discussion

Retinoblastoma is the second most common pediatric malignancy and is a serious threat to children's lives [8]. Retinoblastoma develops mostly under the age of 5, and about 2/3 of children develop the disease before the age of 3 [9, 10]. Timely diagnosis and intervention in the early stages of retinoblastoma results in a survival rate of over 95%, while once extraocular metastases occur, the survival rate is less than 50% [11]. Therefore, in order to achieve early diagnosis and treatment of retinoblastoma, it is increasingly important to find its key genes and biomarkers. Curcumin has antitumor effects on a variety of tumors [12–14]. Curcumin exerts its effects through the downregulation of multiple cellular signaling pathways, including NF-*κ*B, STAT3, activated protein-1, and epidermal growth response-1, all of which are essential for cell development and progression [15]. Yang et al. [16] showed that inhibition of STAT3 phosphorylation contributed to the antiproliferative effect of curcumin on lung cancer cells and inhibited the migration and invasion of cancer cells. Zhang et al. [17] found that curcumin induced endoplasmic reticulum stress in hepatocellular carcinoma BEL-7404 cells by downregulating STAT3 expression, which ultimately promoted apoptosis in BEL-7404 cells. However, the underlying mechanism of curcumin in the treatment of retinoblastoma remains unclear.

In this study, we used network pharmacology and molecular docking to explore the molecular mechanisms of curcumin for retinoblastoma treatment in a more comprehensive manner. We identified three potential targets for curcumin for retinoblastoma treatment through network data mining. GO functional enrichment analysis revealed 517 pathways. KEGG pathway enrichment analysis revealed 94 signaling pathways related to chemical carcinogenesis-receptor activation, chemical carcinogenesis-reactive oxygen species, viral carcinogenesis, Th17 cell differentiation, and other signaling pathways. Molecular docking results showed that curcumin was stably bound to RB1, STAT3, and CDKN2A, among which CDKN2A had the strongest binding to curcumin.

RB1, STAT3, and CDKN2A are the most likely core targets of curcumin for retinoblastoma treatment. Molecular docking analysis has shown that curcumin has a good affinity for these three targets, with CDKN2A showing the highest binding. STAT3 is a well-studied transcription factor in recent years. Several studies have shown that STAT3 has been aberrantly expressed and activated in a variety of tumor tissues and cell lines, can participate in tumor development by inducing cell overproliferation and inhibiting apoptosis, and is aberrantly expressed in retinoblastoma [18, 19]. The RB1 gene is the first family of oncogenes discovered in humans and is an oncogene that regulates the cell cycle, which is closely linked to the development of retinoblastoma [20, 21]. CDKN2A is directly involved in cell cycle regulation and is a novel anticancer gene [22]. Its gene inactivation is closely related to the development of malignant tumors [23]. The main mechanisms include effective inhibition of RNA polymerase activity, alteration of cellular chromatin structure, and prevention of transcription factors from binding to DNA [24]. CNKN2A was found to be differentially expressed in a variety of tumor tissues and showed upregulated expression, which correlated with the pathological characteristics and prognosis of patients [25].

The KEGG enrichment results suggested that the chemical carcinogenesis-reactive oxygen species signaling pathway plays a crucial role, indicating that this signaling pathway is a key link in the treatment of retinoblastoma with curcumin. Reactive oxygen species are produced in the process of oxidative phosphorylation and play an important role in cell and tissue proliferation, differentiation, and apoptosis. Numerous studies have shown that reactive oxygen species are closely associated with the development of retinoblastoma, uveal melanoma, age-related macular degeneration, age-related cataract, dry eye, pterygium, and other ocular-related diseases [26]. Compared with normal cells, the content of reactive oxygen species is higher in tumor cells, and different concentrations of reactive oxygen species have different effects on the development of tumors [27]. Reactive oxygen species not only influence tumorigenesis and development but also play a key role in tumor treatment [27]. Hypoxia promotes the production of reactive oxygen species and activates STAT3 transcription factors, while treatment with reactive oxygen species inhibitors and the antioxidant NAC inhibits STAT3 transcription factor activation, thereby blocking its mediated angiogenic pathway [28]. In the study of Cho et al. [29] on prostate cancer, it was found that that epidermal growth factor promotes prostate cancer cell invasion and metastasis by promoting reactive oxygen species production, which in turn drives STAT3 phosphorylation and regulates the HIF-1*α*/TWIST1/N-cadherin (N-cadherin) signaling pathway. Therefore, STAT3 may be a key target of reactive oxygen species in regulating tumor invasion and metastasis.

## 5. Conclusion

In conclusion, this comprehensive network-based pharmacological analysis suggests a number of testable speculations on the potential molecular mechanisms of curcumin in the treatment of retinoblastoma and predicts RB1, STAT3, and CDKN2A as potential therapeutic targets. This study provides a basis for further experimental studies and ideas to investigate the mechanism of curcumin in the treatment of retinoblastoma, and further studies and validation are needed.

## Figures and Tables

**Figure 1:** The idea and process of this research.

**Figure 2:** Venny analysis diagram of the mapping targets of curcumin and retinoblastoma.

**Figure 3:** GO functional enrichment results of potential targets of curcumin against retinoblastoma.

**Figure 4:** KEGG enrichment results of potential targets of curcumin against retinoblastoma.

**Figure 5:** The protein-protein interaction network among potential targets of curcumin in the treatment of retinoblastoma.

**Figure 6:** Hub genes acquired from the protein-protein interaction network.

**Figure 7:** Modes of docking between curcumin and core targets protein molecules.

**Table 1:** Description of datasets in this study.

Accession	Platform	Experiment type	Tissues	Sample size	References (PMID)
GSE24673	GPL6244	Expression profiling by array	*Homo sapiens*	11	24092970
GSE97508	GPL15207	Expression profiling by array	*Homo sapiens*	9	—
GSE110811	GPL16686	Expression profiling by array	*Homo sapiens*	34	30036517

**Table 2:** Chemical information and binding energy of curcumin.

Mol ID	Chemical abstracts service number	Chemical formula	Molecular weight	Docking protein	Binding energy/(kcal·mol^−1^)
MOL000090	485-37-7	C_21_H_20_O_6_	368.37	RB1	−6.9
				STAT3	−4.8
				CDKN2A	−7.4

## Data Availability

All data used to support the findings of this study are included within the article.
